# A Novel Strategy for the Treatment of Allergic Rhinitis: Regulating Treg/Th17 and Th1/Th2 Balance In Vivo by Vitamin D

This article has been retracted.

**DOI:** 10.1155/2022/9249627

**Published:** 2022-07-31

**Authors:** Baowei Li, Xiaoli Zhang, Zhezhe Sun, Bingxin Xu, Jihua Wu, Hongdan Liu, Haolun Han, Lei Wang, Wei Wu

**Affiliations:** ^1^Department of Otolaryngology, Strategic Support Forces Medical Center, Beijing 100101, China; ^2^Division Two, Strategic Support Forces Medical Center, Beijing 100101, China; ^3^Department of Pathology, Strategic Support Forces Medical Center, Beijing 100101, China

## Abstract

**Objective:**

This prospective study is aimed at observing the number of nasal itching and sneezing in rats from the macroscopic level and examine the pathological changes of nasal mucosa, Th1 and Th2-related cytokines, and Treg/Th17 by vitamin D3 administration from the microscopic level, in order to explore the role of vitamin D in allergic rhinitis and to provide theoretical guidance for prevention and treatment.

**Results:**

There were significant differences in nasal itching and sneezing between the administration groups and the positive groups. Meanwhile, the level of Th1 and Treg in the administration groups increased, while the level of Th2 and Th17 decreased, indicating that the balance of Th1/Th2 was corrected. Our study revealed that vitamin D3 has preventive and therapeutic effects on allergic rhinitis, which provides theoretical guidance for practical application.

## 1. Introduction

It is conservatively estimated that allergic rhinitis (AR) affects more than 500 million people worldwide and has become a health problem affecting humans [1]. Allergic rhinitis is a noninfectious inflammation that includes a group of symptoms, mainly affecting the nasal mucosa [2]. The pathogenesis of allergic rhinitis is not very clear. At present, Th1/Th2 imbalance is considered to be the main cause, and there is no fundamental treatment plan for allergic rhinitis [3–6].

Immunotherapy is considered to be the standard treatment method for long-life relief of symptoms of allergic rhinitis. Recent studies have identified vitamin D as a potential immunomodulator, and it may affect the outcomes of treatment [7–11]. Vitamin D can affect T cells, B cells, monocytes, and macrophages and regulate the activity of DCs. Also, vitamin D can inhibit the differentiation and maturation of DCs in monocytes and downregulate the expression of related stimulatory molecules, thus reducing T cell activity and producing immune tolerance. Vitamin D deficiency can lead to the occurrence of TH2-biased allergic diseases, which may be related to the imbalance of Treg/Th17 cells.

Some studies have shown that the incidence of severe vitamin D deficiency in patients with allergic rhinitis is significantly higher than that normal people, and some studies have shown that children with allergic rhinitis can reduce the symptoms or score of allergic rhinitis by vitamin D-assisted treatment during pollen season. Although there has been some controversy over the efficacy of vitamin D, recent studies have shown a beneficial effect of vitamin D on the course of allergic disease [12–14]. However, many of those studies focused on the symptoms of allergic rhinitis, but the mechanism of vitamin D in curing allergic rhinitis remains unclear.

This study intended to observe the pathological changes of nasal mucosa, Th1 and Th2-related cytokines, and Treg/Th17 changes in sensitized mice through nasal drops and oral administration of vitamin D, so as to explore the causes of vitamin D in the treatment of allergic rhinitis from the micromechanism level and provide theoretical guidance for prevention and treatment.

## 2. Materials and Methods

### 2.1. Materials

Ovalbumin, PMA, and 1A,245-dihydroxyvitamin D3 were obtained from Sigma-Aldrich (St. Louis, MO, USA). Aluminum hydroxide gel, FOXP3 monoclonal antibody, and IL-17 monoclonal antibody were purchased from Thermo Fisher Scientific (Shanghai, China). CD4 monoclonal antibody and CD 25 monoclonal antibody were purchased from Invitrogen (Carlsbad, CA, USA).

### 2.2. Experimental Animals

46 male BALB/c mice weighted 18-20 g in SPF grade were purchased from PLA Strategic Support Characteristic Medical Center. They were randomly divided into 5 groups according to different treatment methods, and each group was randomly divided into two groups once again. All experiments were conducted in accordance with the guidelines of the Institutional Animal Care and Use Committee (IACUC) of PLA Strategic Support Characteristic Medical Center.

### 2.3. Treatment Methods

The mouse allergic rhinitis model was prepared by ovalbumin and aluminum hydroxide [15, 16].

- Suspension preparation: suspension was formed by vibrating mixture of ovalbumin and aluminum hydroxide gel on the oscillator for two minutes. The dose for each mouse is 20 *μ*g ovalbumin in 300 *μ*L aluminum hydroxide gel
- Sensitization stage: 100 *μ*L of newly configured suspension (a total of 300 *μ*L for each) was injected subcutaneously into the abdomen, the left and right back of each mouse on days 1, 8, and 15
- Stimulation stage: since day 22, mice were atomized with 2% OVA solution and inhaled with ultrasonic atomizer for 30 minutes each time for 7 days
- Treatment: 6 mice without any treatment were treated as group 1, 6 allergic rhinitis mice without other treatment were treated as group 2, 8 allergic rhinitis mice treated with vitamin D3 intranasally were named as group 3, anther 8 allergic rhinitis mice treated with vitamin D3 by intraperitoneal injection were named as group 4, and 8 allergic rhinitis mice received PBS injection were considered as group 5. The drug was administered 30 minutes before the C stage of modeling and then atomized again

### 2.4. Nasal Symptoms

The number of sneezes and nasal rubs was counted within 30 minutes of each stimulation since the first stimulation.

### 2.5. Inflammatory Factor Detection

The blood was collected by using a pyrogen- and endotoxin-free test tube and centrifuged at 3000 rpm for 10 min to separate the serum and red blood cells quickly and carefully. The levels of IL-4, IL-5, IL-10, IgE, and INF-*γ* in the supernatant were detected by ELISA kit according to the instructions.

### 2.6. IHC Staining

CD80, CD86, IFN-*γ*, and IL-10 immunoreactivity in nasal mucosa of mice were evaluated by HE and IHC staining. First of all, samples were rehydrated through a process of ethanol for 20 min, 90% ethanol for 2-3 min, 80% ethanol for 2-3 min, and 70% ethanol for 2-3 min. Samples were washed with PBS for 3 times then inactivated by peroxidase at room temperature for 10 min. Then, after washed with PBS, samples were blocked for at 37°C for 1 h. Next, samples were incubated with the primary antibody at 37°C for 2 h and the second antibody 37°C for 1 h in sequence. DAB and hematoxylin were added for 5 min at room temperature according to the order.

### 2.7. Electron Microscopy

Samples were fixed by 4% paraformaldehyde and then immersed in glutaraldehyde at 4°C overnight. After that, samples were soaked in 30%, 50%, 75%, and 90% acetone solution for 10 min according to the order and then soaked in acetone for 5 min (repeated 3 times) for dehydration. After sample preparation, they were observed by TEM.

### 2.8. Statistical Analysis

All data analyses were performed on GraphPad Prism 8.0 software. *P* < 0.05 was considered as a statistical significance.

## 3. Results

### 3.1. Nasal Symptoms

The result of number of nasal itching and sneezing was shown in Table 1. It could be seen that the nasal itching and sneezing number of groups 3 and 4 was significantly different from groups 1, 2, and 5 (*P* < 0.05), while it was almost the same between groups 3 and 4, indicating that intranasal administration may be as effective as intraperitoneal administration.

### 3.2. Inflammatory Factor Detection

As shown in Figure 1, IL-4 and IL-5 levels in group 3 and group 4 were almost the same as group 2 and group 5, while IL-10 level in groups 3 and 4 were slightly higher than that in group 2, which may represent inflammatory factors secretion of Th2, which can promote B cell proliferation and differentiation, induce IgE synthesis, and accelerate respiratory tract remodeling. IFN-*γ* level in group 3 was slightly lower than that in group 5 which indicated that Th1 was slightly downregulated with vitamin D3 administration.

In addition, Treg and Th17 cell markers were tested, and the results showed that CD25+ FOXP3+ level in groups 3 and 4 was higher than that in group 2 while CD4+ IL-17+ level in group 3 was lower than that in group 2. This result suggested that in the vitamin D3 treatment group, the tendency of cell differentiation to Treg cells was enhanced, but the ability to differentiate to Th17 cells was weakened.

### 3.3. IHC Staining

IHC staining showed the intensity of CD-80, CD-86, IFN-*γ*, and IL-10 proteins in nasal mucosa. As shown in Figure 2, the expression of four proteins in mice nasal mucosa showed no significant difference among different groups.

### 3.4. Electron Microscopy

The morphological characteristics of nasal mucosa in different groups were examined by TEM. As shown in Figure 3, the number of intracytoplasmic vacuoles in the nasal mucosal cells of group 2 and group 5 was significantly higher than other groups, indicating the presence of inflammatory response. However, they showed no significant difference between group 1, group 3, and group 4, which mean that administration of vitamin D could inhibit allergic rhinitis in mice.

## 4. Conclusion

Allergic rhinitis is one of the most common pediatric diseases with high incidence worldwide [17–20]. In recent years, the incidence of allergic rhinitis and some respiratory diseases has increased significantly with the aggravation of air pollution and environmental deterioration. Curing allergic rhinitis effectively and safely has attracted more and more attention. To address the problems associated with allergic rhinitis, in this study, we successfully established a model of allergic rhinitis by using a highly sensitive protein, ovalbumin.

Previous studies showed that the level of serum vitamin D (mainly vitamin D 3) in allergic rhinitis patients was generally lower [21–23]. Also, vitamin D was used as immune modulator in a variety of autoimmune diseases [24–26]. However, most previous studies have focused on animal or human macromanifestations to verify the efficacy of vitamin D in the treatment of allergic rhinitis, while the mechanisms has not been thoroughly studied. This may result in limited use of vitamin D. Therefore, in this study, we tested the role of vitamin D3 administration in the development of allergic rhinitis. Patients with allergic rhinitis have increased levels of various proinflammatory factors which also promote disease progression [27, 28]. Our research showed that from the apparent monitoring data, the number of nasal itching and sneezing of groups 3 and 4 (vitamin D3 administration groups) was significantly lower than from groups 2 and 5 (allergic rhinitis group and positive interference group). From a microscopic point of view, the levels of inflammatory factors were assessed. In the vitamin D3 group, the level of IL-10 in groups 3 and 4 was slightly higher than group 2, while the level of IFN-*γ* in group 3 was slightly lower than group 5, indicating that the level of Th1 was increased and the level of Th2 was decreased, resulting in the Th1/Th2-balance corrected [29–32]. Also, in vitamin D3 treatment groups, the tendency of cell differentiation to Treg cells was enhanced, but the ability to differentiate to Th17 cells was weakened [33–35]. Meanwhile, the results of TEM showed that the nasal mucosa of mice in the inflammatory groups showed obvious inflammatory response, while there was no significant difference between the vitamin D3 administration groups and the control group. Although we used two ways of administration in this article, the experimental results showed that there was little difference in the efficacy of oral administration or intraperitoneal injection. Therefore, in our future possible studies, we may focus more on the mechanism behind the efficacy.

In conclusion, vitamin D has been verified to have effect on allergic rhinitis, which can reduce inflammation.

## Figures and Tables

**Figure 1:** Inflammatory factor levels comparison: (a) IL-4, (b) IL-5, (c) IL-10, (d) IFN-*γ*, (e) IgE, (f) CD25+ FOXP3+, and (g) CD4+IL-17+.

**Figure 2:** IHC staining. (a) Nasal tissues from the normal control group (group 1), positive control group (group 2), intranasal administration group (group 3), intraperitoneal injection group (group 4), and positive interference group (group 5). Statistical analysis of CD-80-positive (a), CD-86-positive (b), IFN-*γ*-positive (c), and IL-10-positive (d) staining using ImageJ.

**Figure 3:** Transmission electron microscopy (TEM) images of nasal mucosa.

**Table 1:** Nasal symptoms (*x* ± *s*).

Group	Cases	Nasal itching	Sneeze
1	6	0.3 ± 0.5	0
2	6	11.2 ± 2.6	6.3 ± 0.8
3	8	5.9 ± 0.8	3 ± 0.8
4	8	6.3 ± 0.7	2.6 ± 0.7
5	8	12 ± 1.5	6.5 ± 0.9

## Data Availability

The datasets used and analyzed during the current study are available from the corresponding author upon reasonable request.
